The article "Macrophage-Derived Exosomes in TLR9−/− Mice Ameliorate Sepsis-Induced Mitochondrial Oxidative Stress and Apoptosis in Cardiomyocytes" was retracted in 2023. Reasons: unreliable results or conclusions; concerns about the data; concerns about the peer review; concerns about the citations.

# Macrophage-Derived Exosomes in TLR9^−/−^ Mice Ameliorate Sepsis-Induced Mitochondrial Oxidative Stress and Apoptosis in Cardiomyocytes

**DOI:** 10.1155/2022/5719974

**Published:** 2022-10-03

**Authors:** Xiang Li, Junyu Luo, Yanmei Li, Lu Jia, Yuejin Li, Shili Ye, Lanlan Liu, Yanxuan Yu, Yonggang Lu, Yunpeng Luan

**Affiliations:** ^1^The First Affiliated Hospital of Yunnan University of Traditional Chinese Medicine, Kunming 650021, China; ^2^Department of Life Technology Teaching and Research, College of Life Sciences, Southwest Forestry University, Kunming 650224, China; ^3^The General Surgery Department, The First People's Hospital of Yunnan Province, Kunming 650000, China; ^4^Faculty of Mathematics and Physics, Southwest Forestry University, Kunming 650224, China; ^5^Key Laboratory for Forest Resources Conservation and Utilization in the Southwest Mountains of China, Ministry of Education, Southwest Forestry University, Kunming 650224, China; ^6^Clinical Laboratory, Hebei General Hospital, Shijiazhuang 050000, China

## Abstract

**Objective:**

To explore the mechanisms of TLR9 from macrophages on mitochondrial apoptosis in cardiomyocytes at early stage of sepsis.

**Methods:**

The *in vivo* and *in vitro* sepsis mice were bone marrow transplantation (BMT) with wild type (WT) or (toll-like receptor 9) TLR9 knockout (^−/−^ or KO) myeloid cells and then constructed by cecum ligation and puncture (CLP) as vivo experiment and cardiomyocytes cocultured with WT or TLR9-deficient macrophages treated with LPS as vitro experiment, respectively. Sepsis model were performed by CLP. The expression levels of exosome, PI3K/AKT, and ERK1/2, inflammatory factors, and apoptotic proteins were tested by western blot in vivo. Besides, associated apoptotic proteins and JC-1 fluorescence assay were tested *in vitro*.

**Results:**

The expressions of p-PI3K, p-AKT, exosome markers (CD9, CD63, and TSG101), p-ERK1/2, TNF-*α*, IFN-*γ*, IL-1*β*, and cleaved-caspase-3/-9 were significantly increased in septic mice vs. control mice, and these proteins were declined dramatically in TLR9^−/−^ BMT mice vs. WT BMT mice in sepsis mice models. Meanwhile, the protein expression of cytochrome C, cleaved-caspase-3, and cleaved-caspase-9 increased significantly in primary mouse myocardial cells cocultured with TLR9^−/−^ or WT macrophages stimulated with LPS, and these mitochondrial apoptotic proteins as well as the green 5,5',6,6'-tetrachloro-1,1',3,3'- tetraethylbenzimidazolcarbocyanine iodide (JC-1) fluorescence were dramatically lower in LPS-stimulated cardiomyocytes cocultured with TLR9^−/−^ than with WT macrophages.

**Conclusion:**

TLR9^−/−^ in macrophages suppressed the inflammatory reaction as well as the exosome secretion and resulted in the inhibition of apoptosis and oxidative stress in sepsis-induced cardiomyopathy.

The article "Macrophage-Derived Exosomes in TLR9−/− Mice Ameliorate Sepsis-Induced Mitochondrial Oxidative Stress and Apoptosis in Cardiomyocytes" was retracted in 2023. Reasons: unreliable results or conclusions; concerns about the data; concerns about the peer review; concerns about the citations.

## 1. Introduction

Sepsis, a clinical syndrome with host response disorder caused by infection, is a life-threatening organ dysfunction [1]. It is usually secondary to severe infection, ischemia-reperfusion injury, trauma, and shock [2]. Sepsis often induces varying degrees of cardiac dysfunction, thereby resulting in a poor prognosis [3]. In 1984, Parker et al. [4] discovered reversible cardiac dysfunction in septic patients and proposed the concept of sepsis-induced cardiomyopathy (SIC), the major cause of death in septic patients [5]. To date, the pathogenesis of SIC remains elusive [6], which involves a few of factors such as inflammatory damage, myocardial mitochondrial dysfunction, and oxidative stress injury [7, 8]. Hence, deep exploring the mechanisms of cardiomyocyte injury in sepsis is of important significance for ameliorating the prognosis of sepsis.

During the initiation of sepsis, the obvious change is that monocyte/macrophage injury in patients will cause “endotoxin tolerance,” thus leading to adverse consequences [9]. Monocytes and macrophages are the main components of the innate immune system, which participate in the host's innate immune response by recognizing and presenting antigens, releasing cytokines, and relieving inflammation [10]. However, an excessive immune response may trigger systemic inflammatory response syndrome and compensatory anti-inflammatory response syndrome to protect the human body from sepsis injury. PI3K signal is the major negative and braking mechanism for innate immune reactions. Exosomes are extracellular vesicles secreted by late endosomes; initially, exosomes were considered to be involved in the mechanisms by which reticulocytes transport discarded membrane proteins [11]. Generally, exosomes serve as carriers of informatory molecules that mediate cell-to-cell communication [12]. Macrophage-derived exosomes can participate in innate immune response-induced inflammation through synergistic action with toll-like receptors (TLR) [13]. TLR are regarded as an integral part of the innate immune system [14], among which TLR9 can recognize microbial DNA [15]. Moreover, it has been found that macrophage-derived exosomes can recognize long-chain fatty acids, activate the downstream ERK signaling pathway, and promote the secretion of inflammatory factors [16] and proinflammatory cytokines such as TNF-*α* and L-1*β*, thus inducing the systemic inflammatory cascade response and causing myocardial injury, apoptosis, and cardiac dysfunction [17]. Excessive immune responses are detrimental to the host and negative feedback regulation, and PI3K plays as a primary endogenous suppressor for TLR-induced inflammatory signals in macrophages, which is crucial for the maintenance of immune system as well as cellular structure integrity [18–20]. Previously, much studies were focused on the inflammatory responses and TLR9 signals, whereas the relationship between the PI3K signal-induced exosome secretion and TLR9 activation remains unclear and ambiguous [15, 21]. Therefore, this study was carried on to elaborate on these mechanisms.

The article "Macrophage-Derived Exosomes in TLR9−/− Mice Ameliorate Sepsis-Induced Mitochondrial Oxidative Stress and Apoptosis in Cardiomyocytes" was retracted in 2023. Reasons: unreliable results or conclusions; concerns about the data; concerns about the peer review; concerns about the citations.

In this study, sepsis animal models were constructed in TLR9^−/−^ mice and WT mice by CLP to explore the influencing mechanism of myeloid TLR9 on sepsis-induced inflammatory response *in vivo*, and we also investigate the mechanisms of macrophage-derived exosomes of TLR9^−/−^ mice on sepsis-induced mitochondrial apoptosis in cardiomyocytes *in vitro*.

## 2. Materials and Methods

### 2.1. Experimental Animals and Bone Marrow Transplantation

A total of 48 male C57/BL mice (8-10 weeks old, 22 ± 3 g) were purchased from Beijing Huafukang Biotechnology Co., Ltd. In addition, 48 male C57BL/6J mice (8-10 weeks old, 24 TLR9^−/−^ mice and 24 WT mice) were purchased from the Henan Skbex Biotechnology Company. The TLR9^−/−^ and WT mice were used as donor mice and euthanized with isoflurane, and the myeloid or bone marrow cells were acquired from femur and tibia bones, then the C57/BL mice were irradiated with 5.5 GY, and 6 × 10^7^ donor cells [22, 23] dissolved in RPMI-1640 were injected via caudal veins for the recipient mice. The recipient mice were administrated with acidified water with 100 mg/L neomycin and 10 mg/L polymyxin B sulfate. The BMT animals were placed in a suitable environment at 20 ± 2°C and 55 ± 5% relative humidity, with a 12/12 h light/dark cycle [24]. They had free access to a standard diet and distilled water. The mice BMT with TLR9^−/−^ myeloid cells (TLR9^−/−^ BMT mice) and WT myeloid cells (WT BMT mice) were randomly divided into control and CLP group (subjected to ligation at 1 cm away from the colon end, and the abdominal cavity was closed after two holes were pierced with a 21 gauge needle) and sham operation group (sham group, subjected to laparotomy and cecum exposure, followed by abdominal cavity closure). The heart tissues of mice were sampled and stored at -80°C or 4% paraformaldehyde for subsequent experiments. All studies were approved by the Laboratory Animal Welfare and Ethics Committee.

### 2.2. Extraction and Identification of Exosomes in Sepsis-Cardiomyocyte of Mice

Cardiomyocytes from control or septic mice were ground, and the supernatant fluid was collected and centrifuged at 4°C and 1000 g for 10 min to remove cells and cell debris and then at 4°C and 12000 g for 30 min to remove small particles such as organelles. Later, the supernatant was harvested and filtered by a 0.22 *μ*m filter membrane to remove particles with a size larger than 200 nm. Finally, the filtrate was centrifuged at 4°C and 120000 × *g* for 90 min, and the precipitate obtained after centrifugation was the exosomes. The exosomes were resuspended in PBS buffer (pH = 7.4) and then stored in a refrigerator at -80°C for later use. After the culture is complete, the medium is collected and centrifuged (10,000 × *g*, 30 min, 4°C). The supernatant was then centrifuged at 4°C (110,000 × *g* for 70 min). Wash the precipitate with PBS and centrifuge again at 150,000 *g* for 120 min at 4°C [25]. TEM was used to detect exosome morphology: the exosomes were dropped on a 2 mm copper grid and left for 1 min before adding uranyl acetate staining for 1 min. After drying, the morphology of cellular exosomes was determined by TEM [26].

The article "Macrophage-Derived Exosomes in TLR9−/− Mice Ameliorate Sepsis-Induced Mitochondrial Oxidative Stress and Apoptosis in Cardiomyocytes" was retracted in 2023. Reasons: unreliable results or conclusions; concerns about the data; concerns about the peer review; concerns about the citations.

### 2.3. Isolation and Culture of Bone Marrow-Derived Macrophages

The bone marrow of TLR9^−/−^ mice and WT mice were aseptically harvested in an ultraclean bench, pipetted into a 100 mm^2^ culture dish with 10 mL of induction medium using a sterile syringe, and then pipetted evenly with a pipette tip. On the 3^rd^ day [27, 28], 7 mL of culture supernatant was gently discarded, which was replaced with a fresh induction medium. On the evening of the 6^th^ day, the culture supernatant was discarded and replaced with DMEM containing 10% FBS and double antibody, and the cells were cultured overnight. On the 7^th^ day, after the samples were washed with phosphate-buffered saline (PBS) 3 times, the nonadherent cells were removed, and the macrophages were digested with trypsin for later tests, according to the previous method [29].

### 2.4. Culture and Grouping of Primary Cardiomyocytes

The neonatal mice were collected using sterile tweezers and soaked in 75% alcohol for skin disinfection under a relatively sterile environment. Their hearts were cut into small pieces and rinsed repeatedly with PBS until the rinsing solution was clear. Later, the heart tissues were collected and transferred into a culture flask, which were then added with an appropriate amount of trypsase digest cardiomyocytes for 2-3 minutes, and then left to stand at 4°C overnight. Then, it was added with an appropriate amount of low-glucose DEME complete medium and shaken in a constant temperature water bath box at 37°C at a uniform speed for 5 min. Thereafter, the supernatant was discarded. The tissues were added with 1 mL of collagenase type II and shaken gently in a water bath at 37°C for 30 s, and then, the supernatant was discarded to remove blood cells. Next, 1 mL of collagenase type II was added into the culture flask again. After shaking at 37°C for 15 min in a constant temperature water bath box, the supernatant was collected into a centrifuge tube. The digestion could be repeated many times. After the collected supernatant was centrifuged at 1,000 rpm for 3 min, the supernatant was discarded, and the precipitate obtained was cardiomyocytes. Later, the cell suspension was inoculated into a petri dish and incubated in a 5% CO_2_ incubator at 37°C, and the culture medium was replaced after 24 h, according to the previous method of primary cardiomyocyte culture [30]. Thereafter, the bone marrow-derived macrophages of TLR9^−/−^ mice and WT mice were added into or cocultured with cardiomyocytes, and sepsis-induced cardiomyocyte injury was induced with lipopolysaccharides purchased from Solarbio No. L8880 (LPS: 1 mg/L for 24 h) [31]. The cardiomyocytes were divided into four groups: WT group, TLR9^−/−^ group, WT+LPS group, and TTLR9^−/−^+LPS group.

The article "Macrophage-Derived Exosomes in TLR9−/− Mice Ameliorate Sepsis-Induced Mitochondrial Oxidative Stress and Apoptosis in Cardiomyocytes" was retracted in 2023. Reasons: unreliable results or conclusions; concerns about the data; concerns about the peer review; concerns about the citations.

### 2.5. Western Blotting

Total proteins were extracted from macrophages and cardiomyocytes using radioimmunoprecipitation assay (RIPA) lysis buffer and phenylmethanesulfonyl fluoride (PMSF). The protease inhibitor PMSF was added to fully lyse the cells (PMSF : RIPA = 1 : 100). The cells were centrifuged at 4°C and 12000 g for 15 min. The supernatant was harvested into a 200 *μ*L EP tube and stored at -20°C. The protein concentration in the supernatant was determined using the BCA kit. After SDS-PAGE, the target proteins were transferred onto the PVDF membrane and sealed with 5% skim milk powder at room temperature for 2 h, followed by incubation with primary antibodies (p)-phosphatidylinositol 3-kinase (PI3K), p-protein kinase B (AKT), t-PI3K, t-AKT, cluster of differentiation 9 (CD9), CD63, tumor susceptibility gene 101 (TSG101), p-extracellular signal-regulated kinases 1/2 (ERK1/2), t-ERK1/2, TNF-*α*, IFN-*γ*, IL-1*β*, cytochrome C, cleaved-Caspase-3, Caspase-3, cleaved-Caspase-9, Caspase-9, and GAPDH at 4°C overnight. After that, the membrane was incubated again with HRP-labeled secondary antibodies at room temperature for 2 h. Finally, high-sensitivity ECL kits and the FluorChem Q system were used for exposure, and quantitative analysis of protein was conducted in the AlphaView software.

### 2.6. JC-1 Fluorescence Labeling Assay

After the cells were washed twice with PBS and centrifuged at 2000 g for 5 min, 2 × 10^6^ cells were collected, added with 1 mL of 1 × incubation buffer and 2 *μ*L of JC-1, mixed evenly, and incubated in a 5% CO_2_ incubator at 37°C for 15 min. Later, the supernatant was discarded after centrifugation, and the cells were resuspended with 1 mL of 1 × incubation buffer, followed by detection using a flow cytometer. The above specimens were stained with fluorescence, the different fluorescence colors in 200 cells were observed and counted under a fluorescence microscope, and their percentages were calculated.

The article "Macrophage-Derived Exosomes in TLR9−/− Mice Ameliorate Sepsis-Induced Mitochondrial Oxidative Stress and Apoptosis in Cardiomyocytes" was retracted in 2023. Reasons: unreliable results or conclusions; concerns about the data; concerns about the peer review; concerns about the citations.

### 2.7. Statistical Analysis

CellQuest Pro software was utilized for image analysis, and SPSS 11.5 software was employed for data analysis. The measurement data were expressed as mean ± standard deviation. The experiment was performed 3 times in each group, and the images displayed representative results. One-way ANOVA was used for intergroup comparison, and *t*-test was adopted for comparison between groups. *P* < 0.05 indicated that the difference was statistically significant.

## 3. Results

### 3.1. Myeloid TLR9 Deficiency Improved Structure and Morphology of Myocardium Under Sepsis

Excessive host responses to infection result into sepsis, which induced structural damage of cardiomyocytes and eventually lead to the sepsis-induced cardiac dysfunction, thereby the pathological morphology of cardiomyocytes was firstly observed in this study. We found that in control mice, there were no significant abnormal changes in the heart, mainly exhibited the healthy tissue' morphological structure, whereas in sepsis mice, the WT BMT mice' myocardium showed relatively extensive cellular shrinkage, chromatin condensation, and nuclear fragmentation, and in TLR9^−/−^ BMT mice, these pathological changes were relieved; all these observation indicated that myeloid TLR9 could accelerate the progression of SIC by destroying structures of cell and organelle; all results are shown in Figure 1.

### 3.2. Myeloid TLR9 Knockout Inhibited the Expression of Apoptotic Protein Expressions of Cardiomyocyte in Septic Mice

Cardiomyocytes hardly regenerate and thereby their apoptosis or death is the key and typical characteristics for SIC, and the progression of apoptosis results into the cardiac dysfunction. Prevention of cardiomyocyte death is a pivotal therapeutic strategy for sepsis. In this study, we found in SIC that the myocardial apoptotic proteins of cleaved-caspase-3 and -9 were remarkably increased vs. control groups. Identifying the death or apoptosis was common phenomenon in sepsis-induced cardiac injury. These proteins in TLR9^−/−^ BMT mice cardiomyocytes were significantly decreased compared with WT BMT mice under sepsis inhibited, and all results are shown in Figure 2, which preliminary confirmed the deteriorated effects of myeloid or macrophages' TLR9 in SIC.

### 3.3. TLR9 Deletion Suppressed the Secretion of Exosomes and Activation of the PI3K/AKT in Septic Mice

In the initiation of CLP, PI3K is a powerful inflammation suppressor for avoiding excessive inflammatory response-induced organ damage and dysfunction, and TLR-9 in macrophages is an important inducer for inflammatory responses in sepsis. Therefore, it was found in the CLP experiment that the expressions of p-PI3K, p-AKT, CD9, CD63, and TSG101 in bone marrow-derived macrophages of WT and TLR-9 KO mice increased significantly, while the expressions of t-PI3K and t-AKT were not significantly changed. In the CLP group, the expressions of p-PI3K, p-AKT (Figure 3), and exosome markers (CD9, CD63, and TSG101) (Figure 4) in macrophages of KO mice were significantly lower than those of WT mice, and moreover, the morphology of exosome was observed by TEM, to ensure the exosomes were correctly obtained in this study and shown in S3. In the sham group, there were no obvious differences in the expressions of these proteins between KO mice and WT mice. Considering that the PI3K signal is a primary and powerful promotor for exosome secretion, the findings above indicated that the TLR9 deficiency in macrophages suppresses exosome secretion, which is dependent on its inflammatory inhibition and decreased activation of PI3K signal in sepsis. The suppression of PI3K signal and exosomes in TLR9-deficient mice indicated mild rather than violent inflammation.

The article "Macrophage-Derived Exosomes in TLR9−/− Mice Ameliorate Sepsis-Induced Mitochondrial Oxidative Stress and Apoptosis in Cardiomyocytes" was retracted in 2023. Reasons: unreliable results or conclusions; concerns about the data; concerns about the peer review; concerns about the citations.

### 3.4. TLR9 Deletion Could Repress the Activation of ERK1/2-Induced Inflammatory Factors in Septic Mice

Sepsis is characterized by acute release of multiple inflammatory mediators (such as TNF-*α*, IL-6, and IL-1*β*); excessive release of inflammatory mediators damage tissue and organs. There is increasing evidence that explosive inflammation is associated with cardiac cell death. In innate immune responses, TLR9 is a powerful inducer for the activation of ERK and its downstream inflammatory factors in macrophages, and macrophage-induced inflammation is key for myocardial damage and injury caused by sepsis, thereby the relationship between TLR9-ERK1/2 and inflammatory reactions was next evaluated and studied. Compared with those in the sham group, the expressions of p-ERK1/2, TNF-*α*, IFN-*γ*, and IL-1*β* in macrophages of mice in the CLP group rose significantly, while the protein expression of t-ERK1/2 displayed no evident change. In the CLP group, the expressions of p-ERK1/2, TNF-*α*, interferon-gamma (IFN-*γ*), and IL-1*β* in macrophages of KO mice were significantly lower than those of WT mice, while the protein expression of t-ERK1/2 displayed no marked difference. In the sham group, no significant differences were found in the expressions of these proteins between KO mice and WT mice, as shown in Figure 5. These results indicated that sepsis-induced inflammatory responses in macrophages are largely dependent on the TLR9 signal.

The article "Macrophage-Derived Exosomes in TLR9−/− Mice Ameliorate Sepsis-Induced Mitochondrial Oxidative Stress and Apoptosis in Cardiomyocytes" was retracted in 2023. Reasons: unreliable results or conclusions; concerns about the data; concerns about the peer review; concerns about the citations.

### 3.5. TLR9 Deletion Could Inhibit Myocardial Mitochondrial Apoptosis in Myocardial Tissues of Septic Mice

Apoptosis or death is a salient characteristic of myocardial damage in sepsis, so the relevant indicators were evaluated in sepsis mice. Macrophage-induced inflammation is a major and important factor for myocardial death in sepsis. Compared with those in the sham group, the protein expressions of cytochrome C, cleaved-Caspase-3, and cleaved-Caspase-9 in myocardial tissues of mice in CLP group were significantly increased. In CLP group, the protein expressions of cytochrome C, cleaved-Caspase-3, and cleaved-Caspase-9 in KO mice declined markedly compared with those in WT mice, while the protein expressions of Caspase-3 and Caspase-9 displayed no significant changes. The results indicated that sepsis significantly induces apoptosis and TLR9 deficiency relieves apoptosis or death, which may depend on its inflammatory inhibition.

### 3.6. Macrophages from TLR9^−/−^ Mice Weakened Apoptosis of Primary Cardiomyocytes In Vitro Experiments

The primary cardiomyocytes cocultured with macrophages from WT or TLR9^−/−^ mice were treated with or without LPS to imitate the sepsis cellular model. After LPS stimulation, the protein expressions of cytochrome C, cleaved-Caspase-3, and cleaved-Caspase-9 in mouse cardiomyocytes increased remarkably, while the protein expressions of Caspase-3 and Caspase-9 displayed no obvious changes. Compared with those in the WT+LPS group, the protein expressions of cytochrome C, cleaved-Caspase-3, and cleaved-Caspase-9 in the TLR9^−/−^+LPS group declined dramatically, while the protein expressions of Caspase-3 and Caspase-9 had no significant changes (Figure 6). These results suggested that TLR9 promotes the sepsis-induced myocardial damage or apoptosis, which may depend on the raised level of exosomes carrying inflammatory cytokines.

### 3.7. Variation of Mitochondrial Membrane Potential in Cardiomyocytes In Vitro Experiments

It was observed under the fluorescence microscope that JC-1 formed aggregates in normal cells and emitted orange-red fluorescence. In apoptotic cells, JC-1 existed in the form of monomers and emitted green fluorescence. When the mitochondrial membrane potential is high, JC-1 aggregates in the matrix of mitochondria, forming a polymer that can generate red fluorescence. When the mitochondrial membrane potential is low, JC-1 cannot aggregate in the matrix of mitochondria. At this time, JC-1 is a monomer that can generate green fluorescence. Therefore, the decrease of mitochondrial membrane potential is a landmark event in the early stage of apoptosis. The decrease of cell membrane potential can be easily detected by the change of JC-1 from red fluorescence to green fluorescence. At the same time, the change of JC-1 from red fluorescence to green fluorescence can also be used as an indicator for early apoptosis. After induction with LPS, the number of green fluorescent cells in cardiomyocytes of mice increased, and the *Δψ*m increased. The number of cells emitting green fluorescence declined, and the *Δψ*m decreased in primary cardiomyocytes cocultured with the TLR9^−/−^ macrophages+LPS group compared with those in the WT+LPS group (Figure 7).

The article "Macrophage-Derived Exosomes in TLR9−/− Mice Ameliorate Sepsis-Induced Mitochondrial Oxidative Stress and Apoptosis in Cardiomyocytes" was retracted in 2023. Reasons: unreliable results or conclusions; concerns about the data; concerns about the peer review; concerns about the citations.

## 4. Discussion

As one of the most common critical diseases in clinic, sepsis will induce multiple organ failure, posing a heavy burden on the healthcare system. Starting with infection, this life-threatening disease activates systemic inflammatory response through the production of proinflammatory factors [32]. A cytokine-induced excessive inflammatory response will result in the initial inflammatory “cytokine storm,” which triggers myocardial injury and cardiac dysfunction, dramatically elevating the mortality of patients [33]. The results of this study manifested that (1) TLR9 deletion could inhibit the activation of the PI3K/AKT signaling pathway in bone marrow-derived macrophages of septic mice, thereby suppressing the secretion of exosomes. (2) TLR9 deletion could repress the activation of ERK in bone marrow-derived macrophages of septic mice, thereby reducing the secretion of inflammatory factors. (3) TLR9 deletion attenuated the mitochondrial apoptosis in mouse cardiomyocytes by interfering with the secretion of exosomes from bone marrow-derived macrophages in septic mice.

Myeloid cells mainly and especially the macrophages act as the source of inflammation and direct executor for sepsis. Excessive inflammatory responses are major factors for self-injury in the initiation of sepsis, and the host balance in immune responses especially innate immunity appears particularly important at this stage. Moreover, TLR trigger proinflammatory factor burst by recognizing various bacterial sequences and forming a positive feedback loop. Meanwhile, PI3K is activated as a compensatory negative feedback signal to limit excessive inflammatory signaling [34, 35]. Our findings reflected the overall condition of sepsis-induced injury of cardiomyocytes, and TLR9 deficiency-induced inflammatory inhibition was consistent with the lower activation of PI3K; in other words, a forceful anti-inflammatory mechanism of PI3K is not needed under myeloid TLR-9 deletion in septic cardiomyopathy. Considering that the exosome secretion is mainly modulated by PI3K signals and exosomes act as carriers for extreme inflammatory factors, the suppressed or lowered secretion of exosomes from myeloid macrophages also plays a protective role for sepsis. The activation of PI3K and AKT and the expressions of exosomes CD9, CD63, and TSG101 from WT septic mice increased, and the secretion of macrophage exosomes in TLR9^−/−^ mice was significantly weaker than that in WT mice, which were all found in our in vivo or mouse experiments. In conclusion, myeloid TLR9 deficiency ameliorates inflammatory, strongly implying the mild rather than violent inflammation in sepsis in myeloid TLR9-deletion environments (Figures 3 and 4).

The article "Macrophage-Derived Exosomes in TLR9−/− Mice Ameliorate Sepsis-Induced Mitochondrial Oxidative Stress and Apoptosis in Cardiomyocytes" was retracted in 2023. Reasons: unreliable results or conclusions; concerns about the data; concerns about the peer review; concerns about the citations.

Additionally, combining with sepsis can activate the ERK signaling pathway and promote the secretion of inflammatory factors, thus resulting in inflammatory response [16]. Hence, the activation of ERK and the expressions of inflammatory factors in macrophages in mice were further detected in this study. Our results revealed that the expressions of p-ERK and inflammatory factors TNF-*α*, IFN-*γ*, and IL-1*β* in bone marrow-derived macrophages of KO mice were significantly lower than those in WT mice in sepsis, suggesting that TLR9 deletion can repress the activation of ERK, thereby reducing the inflammatory response. Previous studies focused on TLR-9 and the excessive inflammatory response in cells, such as neutrophils, macrophages, fibroblastic reticular cells, and cardiomyocytes, but the interactions and relationships between two different types of cells in sepsis remain unclear and are urgently needed to clarify [36–39]. This study tried to elaborate on the mechanisms of macrophage TLR-9 in PI3K signal, exosome secretion, inflammatory responses, and myocardial apoptosis in sepsis.

In sepsis, proinflammatory cytokines such as TNF-*α* and IL-1*β* trigger the inflammation cascade, inducing a systemic inflammatory cascade response, which can cause myocardial injury, apoptosis, and cardiac dysfunction [17, 40]. The protein expressions of cytochrome C, cleaved-Caspase-3, and cleaved-Caspase-9 rose remarkably in the myocardial tissues of septic mice, and they were significantly lower in TLR9^−/−^ mice than those in WT mice. Meanwhile, the exosomes from bone marrow-derived macrophages of TLR9^−/−^ mice and WT mice were added into the cardiomyocyte culture medium, respectively, and cardiomyocyte injury was induced with LPS to construct the sepsis models *in vitro*. It was found that in LPS-induced mouse cardiomyocytes, the expressions of mitochondrial apoptosis-related proteins in exosomes from bone marrow-derived macrophages of TLR9^−/−^ mice were significantly lower than those in exosomes from bone marrow-derived macrophages of WT mice, which is consistent with the results of *in vivo* experiments. These results suggested that TLR9 deletion attenuates mitochondrial apoptosis in mouse cardiomyocytes by interfering with the secretion of exosomes from bone marrow-derived macrophages of septic mice. Although new findings about the effects of macrophage TLR-9 on sepsis-induced cardiomyocyte apoptosis were obtained, this study had deficiencies. The living cell workstation can be used to observe the interaction between macrophages and cardiomyocytes from the perspective of space and time analysis, transmission electron microscope can be used to observe the structural changes of subcellular organelles in myocardial cells at different times in sepsis, and the inflammatory data of microfluidic single cell proteome and single-cell intracellular phosphorylation proteomics can be obtained by single-cell proteomics for innate immunologic macrophages of TLR-9^−/−^ mice, which can be used to evaluate and assess the macrophage status in a panoramic state. Moreover, our research may provide the macrophages' TLR-9 levels may be used as a monitoring marker in clinical practice for evaluating the severity of sepsis.

The article "Macrophage-Derived Exosomes in TLR9−/− Mice Ameliorate Sepsis-Induced Mitochondrial Oxidative Stress and Apoptosis in Cardiomyocytes" was retracted in 2023. Reasons: unreliable results or conclusions; concerns about the data; concerns about the peer review; concerns about the citations.

In summary, in early stage of sepsis, TLR9 deletion can inhibit activation of ERK-associated inflammatory responses and meanwhile improved the PI3K/AKT signals as well as exosome secretion, the key regulators for limitation of inflammation, evently resulted into the protective roles SIC.

## Figures and Tables

**Figure 1:** Myeloid deficiency of TLR9 improved morphology of cardiomyocytes in septic mice. (a) WT and TLR9^−/−^ BMT mice in the control group showed health characteristics of cardiac cell structure. (b) TLR9^−/−^ BMT mice improved or inhibited the extensive cellular shrinkage, chromatin condensation, and nuclear fragmentation compared with WT BMT mouse heart. Scar bar: 100 *μ*m.

**Figure 2:** Myeloid deletion of TLR9 suppressed the expression of apoptotic associated proteins in septic mice. (a) The expression of cleaved-caspase-3 and cleaved-caspase-9 of WT and TLR9^−/−^ BMT mice in control and sepsis status. Statistic data of the relative fluorescence intensity of cleaved-caspase-3 and -9 in each group. ^∗^ <0.05 and ^∗∗^ <0.01 vs. septic mice BMT WT myeloid cells.

**Figure 3:** The PI3K signals were lower activated in septic mice BMT TLR9-deficient myeloid cells in early stage of sepsis. (a) The protein levels of phosphorylated and total levels of PI3K and AKT from the heart were WT and TLR9^−/−^ BMT mice in control and sepsis status. (b) Statistic data of western blot were shown. ^∗^ <0.05 and ^∗∗^ <0.01 vs. septic mice BMT WT myeloid cells.

The article "Macrophage-Derived Exosomes in TLR9−/− Mice Ameliorate Sepsis-Induced Mitochondrial Oxidative Stress and Apoptosis in Cardiomyocytes" was retracted in 2023. Reasons: unreliable results or conclusions; concerns about the data; concerns about the peer review; concerns about the citations.

**Figure 4:** The exosome secretion was suppressed in septic mice BMT TLR9-deficient myeloid cells in early stage of sepsis. (a) The exosomes' marker of CD9, CD63, and TSG101 were tested by western blot in WT and TLR9^−/−^ BMT mice of control and sepsis. (b) The statistic data tested by western blot in each group. ^∗^ <0.05 and ^∗∗^ <0.01 vs. septic mice BMT WT myeloid cells.

**Figure 5:** The expressions of ERK-associated inflammatory factors were inhibited in septic mice BMT TLR9-deficient myeloid cells. (a) The cardiac protein levels of phosphorylated levels of ERK1/2 and downstream TNF-*α*, IFN-*γ*, and IL-1*β* as well as the apoptotic associated proteins: cytochrome C and cleaved-caspase-3/-9 were tested by western blot in WT and TLR9^−/−^ BMT mice of control and sepsis groups. (b) The statistic data tested by western blot in each group. ^∗^ <0.05 and ^∗∗^ <0.01 vs. septic mice BMT WT myeloid cells.

**Figure 6:** The apoptotic associated proteins were suppressed in cardiomyocytes cocultured with macrophages' TLR9 deficiency. (a) The protein levels of cytochrome C and cleaved-caspase-3/-9 were tested by western blot in WT and TLR9^−/−^ BMT mice of control and sepsis groups. (b) The statistic data tested by western blot in each group. ^∗^ <0.05 and ^∗∗^ <0.01 vs. primary cardiomyocytes cocultured with WT macrophages.

**Figure 7:** Macrophages' TLR9 deficiency improved cardiomyocytes' mitochondrial membrane potential. (a) The intensity of JC-1 fluorescence in WT and TLR9^−/−^ BMT mice of control and sepsis groups. (b) The statistic data tested by JC-1 staining in each group. ^∗^ <0.05 and ^∗∗^ <0.01 vs. primary cardiomyocytes cocultured with WT macrophages.

## Data Availability

The data used to support the findings of this study are available from the corresponding author upon request.

## Abbreviations

CLP: Cecal ligation and puncture
LPS: Lipopolysaccharides
PI3K: Phosphatidylinositol-3-kinase
AKT: p-protein kinase B
CD9, CD63: Exosome markers
TSG101: Tumor susceptibility gene 101
ERK1/2: p-extracellular signal-regulated kinases 1/2
TNF-*α*: Tumor necrosis factor-alpha
IFN-*γ*: Interferon gamma
IL-1*β*: Interleukin-1 beta
BMT: Bone marrow transplanted
TLR9-/-: Toll-like receptor 9
WT: Wild type
TEM: Transmission electron microscope.
